The article "Meta-Analysis of Matrix Metalloproteinases in the Risk of Cardiovascular and Neurodegenerative Diseases" was retracted in 2024. Reasons: signs of a paper mill; suspected computer-generated content; unreliable results or conclusions; concerns about the data.

# Meta-Analysis of Matrix Metalloproteinases in the Risk of Cardiovascular and Neurodegenerative Diseases

**DOI:** 10.1155/2022/3360316

**Published:** 2022-10-13

**Authors:** Ruizhen Huang, XinYang, Rui Zhu, Junkun Song, Mei Luo, Di-ang Chen

**Affiliations:** ^1^Department of Cardiovascular, Hospital of Chengdu University of Traditional Chinese Medicine, Chengdu, Sichuan 610072, China; ^2^Department of Breast Surgery, Hospital of Chengdu University of Traditional Chinese Medicine, Chengdu, Sichuan 610072, China; ^3^Department of Orthopedics, Nanjing University of Chinese Medicine, Jiangsu 210023, China; ^4^Department of Hospital Infection Management, Hospital of Chengdu University of Traditional Chinese Medicine, Chengdu, Sichuan 610072, China; ^5^Department of Andrology, Hospital of Chengdu University of Traditional Chinese Medicine, Chengdu, Sichuan 610072, China

## Abstract

**Objective:**

To investigate the risk of cardiovascular and neurodegenerative diseases induced by matrix metalloproteinases (MMPs) by meta-analysis.

**Methods:**

Relevant literature was searched from Wanfang Medical Center, CNQI, VIP, PubMed, and other domestic and foreign literature databases for the research direction, and the risk of cardiovascular and neurodegenerative diseases induced by MMPs was meta-analyzed using the fixed-effect model and random-effect model.

**Results:**

MMP-1 and MMP-9 were risk factors for cardiovascular diseases by fixed and random-effect model analysis, respectively, while MMP-2 and MMP-9 were risk factors for increased neurodegenerative diseases by random-effect model analysis.

**Conclusion:**

MMP-1 and MMP-9 are risk factors for cardiovascular diseases, and MMP-2 and MMP-9 are major factors for increased risk of neurodegenerative diseases. MMP-1, MMP-2, and MMP-9 can be used as new targets for clinical diagnosis, treatment, and research of subsequent cardiovascular and neurodegenerative diseases.

## 1. Introduction

Cardiovascular and neurodegenerative diseases are common clinical diseases, with relatively high mortality and morbidity, and is the common pathological mechanism of atherosclerosis that are related to inflammatory and immune reaction; its incidence increased annual outcome for patients with a healthy body and prognosis to cause serious threat. They have become a problem that needs utmost solution in clinical diagnosis and treatment [1, 2].

Matrix metalloproteinases (MMPs) are a superfamily of proteases synthesized and secreted by a variety of cells. These cells include normal tissue cells, inflammatory cells, and tumor cells, whose main function is to degrade extracellular matrix components. It is involved in various physiological and pathological processes such as matrix remodeling and plays an important role in it [3]. It has been clinically verified that MMPs are related to atherosclerosis and inflammatory response and can participate in the pathogenesis of cardiovascular and neurodegenerative diseases through this pathway and have an important impact on the risk of disease occurrence [4, 5]. This study is aimed at determining the effect of MMPs on the risk of cardiovascular and neurodegenerative diseases by using meta-analysis with the help of two statistical models such as the fixed-effect model and random-effect model and by performing heterogeneity test on literature which serves as a basic foundation for successive clinical research and in the treatment of cardiovascular and neurodegenerative diseases (see Figure 1).

## 2. Data and Methods

This section will discuss data retrieval, search criteria, quality evaluation, and statistical methods in detail.

### 2.1. Data Retrieval

The corresponding literatures were searched in the domestic and foreign literature libraries (Wanfang Medical Science, CNKI, VIP, PubMed, etc.) in the direction of “matrix metalloproteinase causes the risk of cardiovascular disease and neurodegenerative disease.” The literature search period was set as January 2007 to May 2022. The key words were matrix metalloproteinases, cardiovascular diseases, neurodegenerative diseases, influencing factors, risks, etc. and a meta-analysis was conducted on the risk of cardiovascular and neurodegenerative diseases caused by matrix metalloproteinases based on the included literatures.

### 2.2. Search Criteria

Inclusion criteria are as follows: (1) in line with the research direction, the research idea was to group the occurrence of cardiovascular or neurodegenerative disease, compare the differences of matrix metalloproteinase index, and analyze the risk of cardiovascular and neurodegenerative disease caused by matrix metalloproteinase index with multivariate logistic regression. (2) The screening conditions do not include gender, nationality, and race. (3) The loss to follow-up rate is less than 20%. (4) All research procedures and operations have been approved by medical research institutions. (5) The literature was published from 2007 to 2022. (6) The data is complete, and there is no obvious loss. (7) There was no obvious operation error in the clinical test of observation indicators. (8) Conform to the research idea of arbitrary screening and observe and analyze any one or more MMP indicators. Exclusion criteria are as follows:(1) the structure of literature content is illogical and repetitive, (2) serious data loss and failure to complete data in an effective way, (3) there is an obvious detection error in any index, (4) basic experiments with cells or animals as research objects, and (5) other research directions or studies do not contain search keywords.

### 2.3. Quality Evaluation

The improved Jadad rating scale was used to evaluate the literature quality. Using this scale, the total score was 1-7, ≤3 was classified as low quality literature, and vice versa.

### 2.4. Statistical Methods

RevMan5.2 statistical software was used for analysis. The count data was expressed as risk ratio (RR), the analysis statistics were expressed as standard mean difference (SMD), and each effect size was expressed as 95% confidence interval (CI). When the heterogeneity between studies was *P* < 0.1 and *I*^2^ ≥ 50%, which was statistically significant, the random-effect model was adopted. The random-effect model is a model used in statistics that uses random variables as model parameters. When the heterogeneity between studies was *P* < 0.1 and *I*^2^ ≥ 50%, then the random-effect model was adopted. In this paper, this model is used because we had obtained the above mentioned results for our dataset. There was no statistical significance in heterogeneity between studies when *P* > 0.1 and *I*^2^ < 50% were satisfied; then, the fixed-effect model was used in the meta-analysis. Clinical and methodological heterogeneity used descriptive analysis.

## 3. Results

### 3.1. Features of Literature Retrieval

A total of 21 Chinese literatures matching the research direction and keywords were screened out after searching the Chinese and English database, including 6 literatures of low quality and 15 literatures of high quality. The basic characteristics and quality evaluation results of the included literatures are shown in Table 1.

### 3.2. Meta-Analysis of Cardiovascular Disease Risk Caused by Matrix Metalloproteinases

#### 3.2.1. Literature Bias on the Risk of Cardiovascular Disease Caused by Matrix Metalloproteinases

A total of 13 Chinese literatures were included on the risk of cardiovascular disease caused by MMP, and the 13 included literatures have no significant publication bias (Figures 1 and 2).

#### 3.2.2. Meta-Analysis of Cardiovascular Disease Risk Associated with MMP-1

Two references were included, and heterogeneity test showed that heterogeneity exists among the references (*I*^2^ = 0.0%, *P* = 0.65). According to fixed-effect model analysis, MMP-1 was associated with a higher risk of cardiovascular disease, and the difference was statistically significant after all studies were combined (OR: 4.39, 95% CI: (2.36, 8.15), *P* < 0.00001). It is suggested that MMP-1 may increase the risk of cardiovascular disease, as shown in Figures 3 and 4.

#### 3.2.3. Meta-Analysis of Cardiovascular Disease Risk Associated with MMP-2

Three references were included, and heterogeneity test showed that there was heterogeneity among the references (*I*^2^ = 0.0%, *P* = 0.98). According to fixed-effect model analysis, there was no significant change in the risk of cardiovascular disease due to MMP-2, and statistically, there was a significant difference observed after all studies were combined (OR: 1.05, 95% CI: (0.80, 1.37), *P* = 0.72). MMP-2 does not increase the risk of cardiovascular disease, as shown in Figures 5 and 6.

#### 3.2.4. Meta-Analysis of Cardiovascular Disease Risk Associated with MMP-9

Eleven articles were included, and heterogeneity test showed that there was heterogeneity among the articles (*I*^2^ = 87.0%, *P* < 0.00001). MMP-9 was associated with a higher risk of cardiovascular disease by random-effect model analysis, with statistically significant differences among studies combined (OR: 1.07, 95% CI: (1.05, 1.09), *P* < 0.00001). MMP-9 may increase the risk of cardiovascular diseases, as shown in Figures 7 and 8.

### 3.3. Meta-Analysis of the Risk of Neurodegenerative Diseases Caused by Matrix Metalloproteinases

#### 3.3.1. Literature Bias on the Risk of Neurodegenerative Diseases Caused by Matrix Metalloproteinases

A total of 8 Chinese literatures were included on the risk of neurodegenerative diseases caused by MMP, and all the 8 literatures included have no significant publication bias (Figures 9 and 10).

#### 3.3.2. Meta-Analysis of the Risk of Neurodegenerative Disease Caused by MMP-2

Two references were included, and heterogeneity test showed that there was heterogeneity among the references (*I*^2^ = 97.0%, *P* < 0.00001). MMP-2 was associated with a higher risk of neurodegenerative diseases by random-effect model analysis, with statistically significant differences between the combined studies (OR: 1.31, 95% CI: (1.15, 1.48), *P* < 0.00001). MMP-2 may increase the risk of neurodegenerative diseases, as shown in Figures 11 and 12.

#### 3.3.3. Meta-Analysis of the Risk of Neurodegenerative Disease Caused by MMP-9

Seven literatures were included, and heterogeneity test showed that there was heterogeneity among literatures (*I*^2^ = 85.0%, *P* < 0.00001). MMP-9 was associated with a higher risk of neurodegenerative disease by random-effect model analysis, with statistically significant differences between the combined studies (OR: 1.01, 95% CI: (1.01, 1.02), *P* < 0.00001). MMP-9 may increase the risk of neurodegenerative diseases, as shown in Figures 13 and 14.

## 4. Discussion

Clinically common cardiovascular and neurodegenerative diseases results in the process of inflammatory reaction and the pathogenesis of atherosclerosis, neurodegenerative diseases on treatment, and prognosis of patients results in severe adverse effects. MMPs participate in a variety of physiological and pathological process that causes cardiovascular and neurodegenerative diseases. And the results of this study showed that MMP-1 is a significant factor for increased risk of cardiovascular disease, but MMP-2 is not a risk factor, which is different from the results of previous studies [27], suggesting that patients with abnormally high expression of MMP-1 are high-risk groups of cardiovascular disease and should be given prior nursing. Based on previous studies, it was believed that the prevalence of cardiovascular diseases is greatly affected by MMP-2. This is due to the fact that MMP-2 and MMP-9 are involved in myocardial development by regulation of the extracellular matrix of myocardium, while MMP-1 and MMP-9 can be brought about by various types of cells such as neutrophiles, fibroblasts, and macrophages to assist in the degradation of cellular matrix constituents and involved in the remodeling process of myocardium via the Ca^2+^ pathway. Also, these matrix metalloproteinases induce the overexpression of fibroblast and growth factor, serves as a stimulus for new connective tissues formation, and ultimately causes cardiovascular injury and diseases such as myocardial fibrosis and irreversible ventricular dilation. There exists a coordinated interaction between matrix metalloproteinases (MMPs) and fibroblast growth factors. MMP-1 and MMP-2 are involved in the transportation of endothelial cells in microvessels (in vitro). Due to the enzymatic action of MMP-1 and MMP-2, fibroblast growth factor is overexpressed and initiates in vitro endothelial cells migration

Perovic et al. [28] believed that MMP-9 can play an important role in the occurrence and development of cardiovascular diseases through multiple pathways such as immunity and inflammation. The results of this study showed that MMP-9 is a significant factor for increased risk of cardiovascular disease, which is basically consistent with the above conclusions, suggesting that the abnormal increase in MMP-9 level can be used as a good reference index for the diagnosis of cardiovascular disease. Analysis of its mechanism is as follows: MMP-9 can be made up of elastin and collagen, gel, and other vascular basement membrane components, plays a role in the degradation of basement membrane, restricts movement, and constricts the smooth muscle cells. MMP-9 through degradation of the vascular basement membrane indirectly impacts the cell wall of vascular smooth muscles, and as a result, membrane in the vascular smooth muscle cells is transferred to the lining and causes proliferation or enlargement. It leads to an increase in extracellular matrix and abnormal proliferation of fibrous tissue, thus causing atherosclerosis and reduced plaque stability thereby increasing the risk of cardiovascular injury. In addition, MMP-9 can promote the development of atherosclerosis and plaque instability by stimulating platelet aggregation, thus increasing the risk of cardiovascular disease [29].

Abe et al. [30] believed that MMPs were overexpressed in patients with Alzheimer's disease (AD) which ultimately caused cognitive dysfunction. This study entails that MMP-2 is a risk factor for neurodegenerative diseases and increases the probability of occurrence of disease, which is consistent with previous results. This suggests the involvement of MMP-2 in the occurrence and development of neurodegenerative diseases that can be used as a new target for subsequent disease prevention, diagnosis, and treatment. One of the familiar example of neurodegenerative diseases is AD, in which Tau protein that is present in nerve cells starts to form tangles from the inner cortex to the hippocampus, edge of the brain, and whole cerebral cortex thus causing severe effects on human cognition. The mechanism of MMP-2 was analyzed from the pathological perspective of AD disease, and MMP-2 was positively correlated with Tau protein. MMP-2 can cut off and decompress the C-terminal of Tau protein without causing significant degradation of highly phosphorylated Tau protein with a pair of helical structure which leads to mass aggregation of the protein and ultimately promoting the occurrence and development of AD [31].

As an important member of the MMP family, MMP-9 is expressed at a low level in the brain tissue and shows an abnormal upward trend in the occurrence of brain injury, AD, and other neurodegenerative diseases. Hoogmartens et al. [32] believed that MMP-9 is highly expressed in patients suffering from cerebral ischemia and brain injury, and patients with a high expression of MMP-9 have a greater proportion of poor prognosis. Similar data were obtained in this study, indicating that MMP-9 can increase the clinical risk of neurodegenerative diseases, and this indicator is an independent risk factor for neurodegenerative diseases. The reasons are as follows: Combined with the pathological research results of cerebral ischemia and brain injury, it is verified that atherosclerosis is the main pathological mechanism of the disease, plaque rupture, and blood flow disorder will increase the risk of the disease. MMP-9 is a very sensitive inflammatory indicator that can reflect the active state of atherosclerosis in real time and is a key enzyme protein of collagen degradation. For the degradation of collagen, it plays a vital role by degrading the fibrous cap. Abnormally elevated levels of MMP-9 cause degradation of a large number of fibrous caps and thickness contraction, cause erratic plaques directly, and also provoke rupturing of plaque thereby promoting the hyperactivity of coronary atheroschlerosis; all these conditions ultimately result in neurodegenerative diseases such as brain ischemia and injury. In addition, MMP-9 is a proinflammatory protease, and its abnormally high expression can cause destruction in the basal membrane of cerebrovascular wall, thereby increasing and damaging the permeability of the blood-brain barrier (BBB) in the body, and ultimately causing brain injury [33].

In the design of this study, only three MMP indicators, MMP-1, MMP-2, and MMP-9, were included in the outcome index for observation, and there were only a small number of included literatures and lack of English literatures. All these deficiencies may increase the overall data bias of the study.

## 5. Conclusion

In short, three matrix metalloproteinases have been studied in this article and it was observed that MMP-1 and MMP-9 are risk factors for cardiovascular diseases according to fixed-effect model while MMP-2 and MMP-9 are risk factors for increased risk of neurodegenerative diseases according to the random-effect model. MMP-1, MMP-2, and MMP-9 can be used as novel targets for the prevention, diagnosis, and treatment of cardiovascular and neurodegenerative diseases.

## 6. Future Prospects

In this study, the risk of cardiovascular disease and neurodegenerative disease caused by matrix metalloproteinases is taken as the entry point. Other MMP observational indicators can be added in subsequent studies, and on this basis, the risk of cardiovascular disease and neurodegenerative disease caused by MMP gene polymorphism is taken as the direction of in-depth analysis.

## Figures and Tables

**Figure 1:** Overall literature bias of MMP-induced cardiovascular disease risk.

**Figure 2:** Overall literature bias of MMP-induced cardiovascular disease risk.

**Figure 3:** Metaforest map of cardiovascular disease risk associated with MMP-1.

**Figure 4:** Metafunnel plot of MMP-1 for cardiovascular disease risk.

**Figure 5:** Metaforest map of cardiovascular disease risk associated with MMP-2.

**Figure 6:** Metafunnel plot of MMP-2 associated with cardiovascular disease risk.

**Figure 7:** Metaforest map of cardiovascular disease risk associated with MMP-1.

**Figure 8:** Metafunnel plot of MMP-1 for cardiovascular disease risk.

**Figure 9:** Overall literature bias on the risk of neurodegenerative diseases caused by MMP.

**Figure 10:** Overall literature bias on the risk of neurodegenerative diseases caused by MMP.

**Figure 11:** Metaforest map of the risk of neurodegenerative diseases caused by MMP-1.

**Figure 12:** Metafunnel plot of the risk of neurodegenerative disease caused by MMP-1.

**Figure 13:** Metaforest map of the risk of neurodegenerative diseases caused by MMP-1.

**Figure 14:** Metafunnel plot of the risk of neurodegenerative diseases caused by MMP-1.

**Table 1:** Literature retrieval information and quality score.

Document	Outcome indicators	Published time	Quality score
Cheng et al. [6]	②③	2019	4
Li et al. [7]	③	2019	4
Li et al. [8]	③	2016	3
Ma et al. [9]	②	2007	2
Ma et al. [10]	③	2018	4
Qin [11]	③	2014	3
Teng et al. [12]	③	2021	4
Wang et al. [13]	③	2014	3
Wei et al.[14]	③	2018	4
Xu and Deng [15]	①②③	2015	6
Zhou and Liu [16]	③	2020	4
Zhao et al. [17]	①	2020	4
Zhou et al. [18]	③	2020	4
Mondian et al. [19]	②③	2016	5
Fan et al. [20]	③	2021	4
Hou et al. [21]	③	2022	4
Wang et al. [22]	③	2018	4
Wang et al. [23]	③	2021	4
Wang et al. [24]	③	2017	4
Yan et al. [25]	②	2017	3
Yue et al. [26]	③	2014	3

Notes: ① MMP-1, ② MMP-2, ③MMP-9.

## Data Availability

The datasets used in this paper are available from the corresponding author upon request.

## References

[1] Selejan S. R., Hewera L., Hohl M. (2017). Suppressed MMP-9 activity in myocardial infarction-related cardiogenic shock implies diminished rage degradation. *Shock*.

[2] Fu N., Li H., Sun J., Xun L., Gao D., Zhao Q. (2018). Trichosanthes pericarpium aqueous extract enhances the mobilization of endothelial progenitor cells and up-regulates the expression of VEGF, eNOS, NO, and MMP-9 in acute myocardial ischemic rats. *Frontiers in Physiology*.

[3] Beroun A., Mitra S., Michaluk P., Pijet B., Stefaniuk M., Kaczmarek L. (2019). MMPs in learning and memory and neuropsychiatric disorders. *Cellular and Molecular Life Sciences*.

[4] SoukhakLari R., Moezi L., Pirsalami F., Moosavi M. (2018). The effect of BSA-based curcumin nanoparticles on memory and hippocampal MMP-2, MMP-9, and MAPKs in adult mice. *Journal of Molecular Neuroscience*.

[5] Zhou L., Kou D. Q. (2019). Correlation between acute myocardial infarction complicated with cerebral infarction and expression levels of MMP-2 and MMP-9. *European Review for Medical and Pharmacological Sciences*.

[6] Cheng Y. L., Chen J., Chen H. Y., Tuo T., Liu D. (2019). Serum soluble ST2, matrix metalloproteinase 2 and matrix metalloproteinase 9 levels and their relationship with cardiovascular events in patients with chronic heart failure. *Journal of Applied Cardio-Cerebral Pulmonary Vascular Diseases*.

[7] Li B. L., Su H., Ma J. S., Li M., Geng L. (2019). Expression of depolymerin-like metalloproteinases in oxidized low density lipoprotein (LDL-C) and platelet-binding protein (PLATelet-binding protein i) mods and their relationship with coronary plaque stability in patients with acute myocardial infarction. *Chinese Journal of Clinical Pharmacology*.

[8] Li N., Lu J. H., Dai X. Y. (2016). Correlation between metalloproteinase-9 and prognosis in patients with acute coronary syndrome. *Journal of Clinical Emergency*.

[9] Ma T., JXg W., Sun X. (2007). Serum levels of C-reactive protein, soluble CD40 ligand and matrix metalloproteinase-2 in patients with coronary heart disease. *Journal of Clinical Cardiology*.

[10] Ma W. L., Zhang Y. L., Bao F. M., Cai Y. (2018). Correlation of plasma matrix metalloproteinase-9 with h-type hypertension and coronary artery disease. *Chinese Journal of Evidence-Based Cardiovascular Medicine*.

[11] Qin X. I. H. (2014). Relationship between matrix metalloproteinase-9 and its inhibitors and carotid atherosclerosis in elderly with hypertension. *Guangxi Medical Journal*.

[12] Teng L. F., Lin J., Liu S. W., Ye C., Qiao P., Wang Y. (2021). Relationship between expression of serum adipocytokine Apelin and matrix metalloproteinase-9 and arrhythmia after acute myocardial infarction. *Journal of Clinical Military Medicine*.

[13] Wang K. K., Qin Q., Li Y. (2014). The relationship between homocysteine and matrix metalloproteinase 9 and coronary heart disease. *Clinical Meta-Clin*.

[14] Wei N., Li Z., Chen J., He J. (2018). The role of high sensitivity C-reactive protein, matrix metalloproteinase-9 and carotid plaque stability in predicting cardiac events in acute coronary syndrome. *Ningxia Medical Journal*.

[15] Xu Y. Q., Deng W. (2015). Relationship between matrix metalloproteinases, osteopontin, cTnI, cTnT and ventricular remodeling in patients with heart failure. *Lingnan Journal of Cardiovascular Disease*.

[16] Zhou L., Liu H. B. (2020). Correlation analysis of microangiopathosis and endothelin, matrix metalloproteinase-9 and other risk factors in elderly type 2 diabetes mellitus. *Journal of Practical Medicine*.

[17] Zhao Z. K., Zhai H., Li L., Liu R., Xia Y. (2020). Relationship between tumor necrosis factor -*α* and matrix metalloproteinase-1 and ventricular remodeling in elderly patients after myocardial infarction. *Hebei Medicine*.

[18] Zhou F. L., Zhu Z. Z., Lu L. (2020). Coronary artery calcification and its correlation with serum galactolectin 3 and matrix metalloproteinase 9 levels in patients with maintenance hemodialysis. *Guangxi Medical*.

[19] Mondian Z., Wang X., Wang H. F., Zhuang S., Xing M. (2016). Serum MMP-2 and MMP-9 levels in patients with Alzheimer’s disease and mild cognitive impairment. *China Medical Journal*.

[20] Fan Y. H., Liu H. Q., Li W. F., Lv S., He X., Li X. (2021). Analysis of the levels of VILIP-1, MMP-9 and Apo E in patients with vascular dementia. *Journal of Practical Clinical Medicine*.

[21] Hou W. Z., Liu S. H., Zhong P. (2022). Study on the relationship between matrix metalloproteinase-3 and matrix metalloproteinase-9 in ischemic white matter lesions. *Journal of Anhui Medicine*.

[22] Ni M., Yu F., Wang Y. (2021). Correlation between matrix metalloproteinase-9 and transient ischemic attack prognosis. *Journal of Clinical And Experimental Medicine*.

[23] Wang C., Xie J., Luo S., Ye M., Shi P., Liu D. (2021). Correlation between matrix metalloproteinase-9 and transient ischemic attack prognosis. *Journal of Clinical and Experimental Medicine*.

[24] Wang F., Ni J., Zhou Y., Jiang M., Sha D. (2017). Prediction of serum matrix metalloproteinase-9 and ferritin in patients with acute ischemic stroke. *International Journal of Cerebrovascular Disease*.

[25] Yan S. J., Piao X. Y., Zhao J., Liang Q. (2017). Expression of matrix metalloproteinase-2 in brain MRI of patients with white matter lesions. *Journal of Clinical Neurology*.

[26] Yue Y. H., Bai X. D., Zhang X. N. (2014). Serum level and gene of matrix metalloproteinase 9-1562C>T polymorphism and clinical classification of acute ischemic stroke in uygur. *Chinese Journal of Arteriosclerosis*.

[27] Fernandez Machulsky N., Gagliardi J., Fabre B. (2016). Matrix metalloproteinases and psychosocial factors in acute coronary syndrome patients. *Psychoneuroendocrinology*.

[28] Perovic M., Obradovic M., Resanovic I., Isenovic E. R. (2018). Editorial: relationship between vitamin D and metalloproteinases (MMPs) in acute myocardial infarction (AMI). *Current Vascular Pharmacology*.

[29] Bertelsen D. M., Neergaard J. S., Bager C. L. (2018). Matrix metalloproteinase mediated type I collagen degradation is an independent predictor of increased risk of acute myocardial infarction in postmenopausal women. *Scientific Reports*.

[30] Abe K., Chiba Y., Hattori S. (2020). Influence of plasma matrix metalloproteinase levels on longitudinal changes in Alzheimer's disease (AD) biomarkers and cognitive function in patients with mild cognitive impairment due to AD registered in the Alzheimer's Disease Neuroimaging Initiative database. *Journal of the Neurological Sciences*.

[31] Biswas M. H. U., Almeida S., Lopez-Gonzalez R. (2016). MMP-9 and MMP-2 contribute to neuronal cell death in iPSC models of frontotemporal dementia with *MAPT* mutations. *Stem Cell Reports*.

[32] Hoogmartens J., Hens E., Engelborghs S. (2021). Investigation of the role of matrix metalloproteinases in the genetic etiology of Alzheimer’s disease. *Neurobiology of Aging*.

[33] Zhang D., Jie Z. B. (2020). Expression and clinical significance of matrix metalloproteinase-9 and hypoxic inducer factor-1 *α* in patients with ischemic stroke in plateau area. *International Journal of Neurology and Neurosurgery*.

